The article "Correlation of Serum FGF23 and Chronic Kidney Disease-Mineral and Bone Abnormality Markers With Cardiac Structure Changes in Maintenance Hemodialysis Patients" was published in 2023. Journal: Evid Based Complement Alternat Med.

# Correlation of Serum FGF23 and Chronic Kidney Disease-Mineral and Bone Abnormality Markers With Cardiac Structure Changes in Maintenance Hemodialysis Patients

**DOI:** 10.1155/2023/6243771

**Published:** 2023-04-08

**Authors:** Dewang Zeng, Aiyun Zha, Ying Lei, Zongchao Yu, Rui Cao, Ling Li, Zhuoheng Song, Weilong Li, Yunyi Li, Haiping Liu, Shaoxing Huang, Xiangnan Dong, Bernhard Krämer, Berthold Hocher, Lianghong Yin, Chen Yun, Stanislao Morgera, Baozhang Guan, Yu Meng, Fanna Liu, Bo Hu, Shaodong Luan

**Affiliations:** ^1^Department of Nephrology, The First Affiliated Hospital of Jinan University, Jinan University, Guangzhou, China; ^2^Department of Nephrology, Huadu District People's Hospital, Guangzhou, China; ^3^Hospital of South China Agricultural University, Guangzhou 510642, China; ^4^Department of Nephrology, Shenzhen Longhua District Central Hospital, Guangdong, Shenzhen 518110, China; ^5^The Second People's Hospital of Lianping County, Heyuan, Guangdong 517139, China; ^6^Fifth Department of Medicine, University Medical Centre Mannheim, University of Heidelberg, Mannheim, Germany; ^7^Department of Nephrology, Charité -Universitätsmedizin Berlin, Campus Mitte, Berlin, Germany

## Abstract

**Background:**

CKD-MBD is a mineral and bone metabolism syndrome caused by chronic kidney disease. FGF23 is an important factor regulating phosphorus and is the main influencer in the CKD-MBD process. In this study, we observed the correlation among serum FGF23 and calcium, phosphorus and parathyroid hormone, and the correlation between FGF23 levels and cardiac structural changes in MHD patients.

**Methods:**

We examined serum FGF23 concentrations in 107 cases of MHD patients using the ELISA method, recorded demographic information and biochemical data, and analyzed the correlation between serum FGF23 levels and blood calcium and blood phosphorus and PTH levels. All patients were evaluated by cardiac color ultrasound, and we finally analyzed the association between the FGF23 level and cardiac structural changes.

**Results:**

In 107 cases of MHD patients, serum FGF23 levels were linearly associated with serum calcium (*r* = 0.27 *P* < 0.01) and parathyroid hormone levels (*r* = 0.25, *P* < 0.05). FGF 23 was negatively correlated with age (*r* = −0.44, *P* < 0.01).Serum FGF23 levels were correlated with right atrial hypertrophy in HD patients (*P* < 0.05). No correlation was found among FGF23, left ventricular hypertrophy/enlargement, and valve calcification stenosis (*P* > 0.05).

**Conclusion:**

Serum FGF23 showed a positive correlation among blood calcium levels and PTH levels in hemodialysis patients, and FGF23 levels can affect the incidence of right atrial hypertrophy in MHD patients.

## 1. Introduction

Chronic kidney disease (CKD) is a serious disease threat to human health, and cardiovascular complications are the leading cause of death in CKD patients [1]. However, how to delay the progression of chronic kidney disease as well as how to reduce the risk of cardiovascular outcomes are still major challenges in nephrology [2]. Chronic kidney disease-mineral and bone abnormalities (CKD-MBD) is a syndrome of abnormal mineral and bone metabolism caused by chronic kidney disease, including abnormal calcium and phosphorus metabolism, parathyroid hormone (PTH) changes, and bone mineralization, and reduced bone mass and osteomalacia [3, 4]. Fibroblast growth factor 23 (FGF23) is an important phosphate metabolism regulator secreted by osteocytes. It inhibits phosphorus reabsorption through renal tubules and suppresses parathyroid hormone secretion and the synthesis of active vitamin D3, thus limiting phosphate absorption in the intestine [5, 6]. Several studies showed FGF23 was independently associated with left ventricular hypertrophy, and there were many observational clinical reports on the positive correlation between FGF23 and vascular calcification in CKD patients [7]. How does FGF23 influence the cardiac structural changes in hemodialysis patients is our concern.

A longitudinal study indicates that increased FGF23 is linearly associated with mortality in hemodialysis patients [8]. Accumulating recent clinical evidence suggests that FGF-23 plays a regulatory role in multiple pathological processes in cardiovascular diseases, such as coronary atherosclerosis, vascular calcification, left ventricular hypertrophy, and myocardial injury [7, 9, 10]. Conversely, another investigation establishes that FGF23 is not associated with arterial calcification [11]. The correlation between FGF23 levels and altered cardiac structure and indicators of disturbed mineral and bone metabolism in hemodialysis patients is not clear. This cross-sectional observational study aims to explore the correlation between serum FGF23 levels and mineral and bone abnormalities in hemodialysis patients, as well as to assess any potential correlations with cardiac structural changes in hemodialysis patients. In addition, we investigate FGF23 as the potential biomarker of adverse cardiovascular outcomes in hemodialysis patients.

## 2. Methods

### 2.1. Study Population

In this retrospective, single-center, observational study, 107 maintenance hemodialysis (MHD) patients (58 males and 49 females) in the Hemodialysis Center of Huadu District People's Hospital in Guangzhou (China) were selected for participation from September 2018 to December 2019. Of these patients, 42 were with chronic glomerulonephritis, 29 with diabetic nephropathy, 14 with hypertensive renal impairment, 7 with gout nephropathy, 5 with obstructive nephropathy, 6 with polycystic kidney, and 4 with lupus nephritis. The following inclusion criteria were applied: diagnostic criteria for CKD stage 5 were met and MHD was received for >three months. The exclusion criteria employed were as follows: the use of immunosuppressants within the present month; history of severe infection in the recent March or surgery or trauma within the present month; severe malnutrition or malignant tumors; and patients unable to undergo cooperative examination. This clinical study was reviewed and approved by the hospital Ethics Committee (no. 2022007), and all the patients participating in the project signed the informed consent form.

### 2.2. Clinical Data Collection

We collected the basic clinical information of all patients, including age, gender, dialysis age, primary disease, and accompanying disease. Patients' laboratory examination results, including serum creatinine (sCr), blood urea nitrogen (BUN), hemoglobin (Hb), albumin (Alb), calcium (Ca), phosphorus (P), parathyroid hormone (PTH) value, and other indicators, were also collected.

### 2.3. Measurement of Serum FGF23

Blood samples were collected before hemodialysis, and the serum fluid was collected by centrifugation. The serum FGF23 levels were measured by enzyme-linked immunosorbent assay (ELISA). The human FGF23 ELISA kits utilized in this study were manufactured by Immutopics International (San Clemente, CA, USA; #60–6600).

### 2.4. Cardiac Color Ultrasound Evaluation

All MHD patients underwent doppler color ultrasound for evaluation of the cardiac structure and function using the Philip company doppler ultrasound instrument. Doppler color ultrasound examination measured the patient's right atrial diameter (RA), left atrial diameter (LA), left ventricular posterior wall thickness (LVPW), pulmonary artery diameter (PA), right chamber diameter (RV), left ventricular contraction fraction (FS), left ventricular ejection fraction (LVEF), and the values of other parameters.

### 2.5. Statistical Analysis

SPSS 21.0 statistical software was used for statistical analysis. Measurement data conforming to normal distribution were expressed as mean ± standard deviation, whereas nonnormal distribution data were presented as median and quartiles. The *t*-test was implemented to determine the means of normal distribution data between the two groups. For count data, we used frequency and ratio, and for group comparison, we conducted a chi-square test. Correlation analysis was next performed using the Pearson correlation analysis method. *P* < 0.05 was considered to indicate statistically significant differences.

## 3. Results

### 3.1. Clinical Baseline Characteristics of the MHD Patients

The mean age of the MHD patients was 57.5 ± 14.3 years. A total of 58 (54.2%) males and 49 (45.8%) females were enrolled in the study. The mean dialysis time was 50.8 ± 33.7 months. The detailed baseline information of the biochemical indexes, including Hb, Alb, sCr, BUN, uric acid (UA), TG, CHOL, LDL, HDL, Ca, P, PTH, and FGF23 levels of all MHD patients are displayed in Table 1.

Twenty-eight healthy volunteers were selected for measurements of FGF23. The mean FGF23 value in healthy controls was 17.14 ± 6.64 (pg/mL), whereas in MHD patients, it was significantly higher compared with healthy controls, with *t* = −9.093 and *P* < 0.01.

The analysis of the Pearson correlation between FGF23 levels and those of age, calcium, phosphorus, and PTH.

Table 2 indicates the Pearson correlation analysis between the levels of FGF23 and the ones of Ca, P, and PTH. After multivariate linear regression analysis for FGF23, we found that Age and PTH, calcium were the factors related to FGF23 levels. Serum FGF23 had a negative linearly correlation with age (*r* = −0.44, *P* < 0.001), serum FGF23 had a positive linearly correlation with blood calcium (*r* = 0.27, *P* = 0.005); and serum FGF23 had a positive linearly correlation with serum PTH levels (*r* = 0.25, *P* = 0.01), see Tables 2 and 3, Figure 1).

Comparison of the clinical data and biochemical indexes among the different FGF23 level groups.

Grouping was performed according to the FGF23 horizontal line quartile method. Group 1: FGF23: (3.75–172.03) pg/mL, *N* = 25 cases; Group 2: FGF23: (182.13–1146.13) pg/mL, *N* = 26 cases; Group 3: FGF23: (1186.17–6314.80) pg/mL, *N* = 27 cases; and Group 4: FGF23: (6438.10–14, 610.14) pg/mL, *N* = 29 cases. The comparison of clinical data and biochemical indicators between the groups with different FGF23 levels are presented in Table 4 and Figure 2.

By FGF23 quartile grouping analysis, with the increased level of serum FGF23, the levels of serum calcium, serum inorganic phosphorus, and PTH showed a linear increase tendency. There is a significant difference between group 2 and group 4 in serum calcium levels (*P*=0.033), there is a significant difference between group 1 and group 4 in PTH levels (*P*=0.044).

Comparison of clinical Cardiac ultrasound parameters among different FGF23 concentration groups (see Table 5).

There is a significant difference among group 3 and group 1 or group 2 in the right atrial enlargement ratio (*P* < 0.05).

## 4. Discussion

Currently, there are nearly 10%–15% of adults affected by CKD worldwide, making it a considerable burden for public health [12]. CKD-MBD represents a major clinical complication in patients with chronic renal disease MHD and is an important factor affecting survival and mortality. Discovered recently, FGF23 is a core factor regulating the bone and mineral metabolism axis; higher concentrations can be detected in the serum of early-stage CKD patients [13]. In addition, FGF23 was found to be a major risk factor for cardiovascular events in CKD patients [14]. Nevertheless, the association between FGF23 and cardiovascular complications has not been assessed in CKD-MBD patients.

In this study, we found that the mean FGF23 level in CKD-MBD patients was significantly higher than that in healthy controls (*P* < 0.05). The general increase in FGF23 is an important factor in the development of CKD-MBD in MHD patients. FGF23 is a hormone secreted by osteogenic cells, which is involved in the suppression of osteoblast differentiation, proliferation, and activation, thereby inhibiting bone mineralization.

The level of FGF23 was increased in early-stage CKD patients, which was identified as the earliest regulator of calcium, phosphorus, and bone metabolism, involved in phosphorus homeostasis maintenance [15]. Further analysis found that in MHD patients with different FGF23 level groups, the serum calcium, serum phosphorus, and PTH increased linearly with the elevation in the FGF23 levels. Furthermore, statistically significant differences were established in the blood calcium and PTH among the different FGF23 groups (*P* < 0.05). Another study showed that PTH increased the expression of the FGF23 gene [16]. Thus, we speculate that controlling blood calcium levels and reducing PTH concentration can lower the level of FGF23, and thus regulate the “master switch” of CKD-MBD development. In addition, considering the FGF23 values increased significantly with the progression of hyperphosphatemia, the use of phosphorus binders is a necessary treatment of CKD-MBD. New phosphorus binders such as sevelamer hydrochloride and lanthanum carbonate were recommended. Sevelamer hydrochloride has shown to reduce the serum FGF23 levels in CKD patients and CKD patients on dialysis [17, 18]. Lanthanum carbonate also reduced the FGF23 level in CKD patients [19].

Interestingly, in this study, we found that increased serum uric acid was also significantly associated with elevated FGF23. Serum uric acid levels were significantly increased between group 2 and group 4 (*P* < 0.05). An earlier study discovered that hyperuricemia was associated with the occurrence of cardiovascular events in CKD patients [20]. Therefore, we assumed that hyperuricemia contributed to the acceleration of CKD-MBD progression.

To explore the association factors between FGF23 and the occurrence of cardiovascular events in MHD patients, we further investigated the cardiac structure and performed functional evaluation in MHD patients. We found that the incidence of LV hypertrophy in early-to-final-stage CKD patients was within 50%–90%, which is the most important factor aggravating cardiovascular events in CKD patients [21]. A previous study indicated that high FGF23 levels are independent predictors of LV hypertrophy in CKD [22]. In this investigation, we established that the incidence of LV hypertrophy and LV enlargement in MHD patients reached 56.0% and 23.3%, respectively. However, no significant difference was found between the groups with different levels of FGF23, and there was no significant intergroup difference in the left ventricular ejection fraction (LVEF) (*P* > 0.05). In CKD-MBD, the abnormal deposition of calcium and phosphate in the blood vessels, valves, and the heart leads to vascular calcification. An earlier clinical study showed that vascular calcification was an independent predictor of increased cardiovascular mortality in patients with CKD [23]. Cardiac valve calcification and stenosis are common factors leading to decreased cardiac function and a common manifestation of CKD-MBD. Here, the incidence of cardiac valve stenosis in MHD patients was also very high, reaching 45.7%, with no significant intergroup difference in the FGF23 concentration (*P*=0.351). We also found significant intergroup variations in the rate of the right atrial enlargement; the high‐concentration group 3 had a higher incidence level than the low-concentration group 1. These results suggest the presence of an association between the FGF23 concentration and the enlargement of the right atrium, which may be related to the stenosis of the tricuspid valve, so the calcification/stenosis of the valve can lead to enlargement of the right chamber.

In addition, we are also concerned that abnormal lipid metabolism such as hyper-LDL-emia in MHD patients also increased with the rise in the FGF23 levels. The findings of some studies pointed out a positive relationship between blood FGF23 and LDL in patients with coronary heart disease [24]. Similarly, in the current study we found that the increased LDL levels accompanied by the serum FGF23 concentration elevated in MHD patients. In the present study, the increase in HDL was significantly higher in the high-concentration FGF23 group 4 (*P* < 0.05). We suggest that lipoprotein abnormalities also play an important role in the increase of FGF23 in MHD patients.

This single-center cross-sectional retrospective study has some limitations. First of all, the sample size was small, and the results were representative only of our dialysis center group. A randomized controlled clinical study with large samples is needed to further explore the association of high FGF23 levels with clinical complications and biochemical indicators in MHD patients. Second, the direct correlation between high FGF23 levels and cardiovascular events in HD patients was not explored here and is to be the direction of our subsequent research work.

## 5. Conclusions

In conclusion, in the present study, we conducted a research study into the clinical aspects and features of hyper-FGF23-emia in MHD patients. We found that FGF 23 was positively correlated with PTH (*r* = 0.25, *p*=0.010) and calcium (*r* = 0.27, *p*=0.005), but was no statistical correlation with phosphate. FGF 23 was negatively correlated with age (*r* = -0.44, *p* < 0.0001). FGF23 was positively correlated with right atrial hypertrophy. No correlation was found among FGF23, left ventricular hypertrophy/enlargement, and valve calcification stenosis (*P* > 0.05). Therefore, hyper-FGF23-emia is a clinical phenomenon that requires continuous attention from nephrologists and hemodialysis physicians and may be a key tool for early intervention in achieving improvement in CKD-MBD patients.

## Figures and Tables

**Figure 1:** The correlation of FGF23 with PTH (a), Ca (b), and age (c).

**Figure 2:** Comparison of PTH, Ca, and *P* value among FGF23 groups.

**Table 1:** Baseline clinical and laboratory characteristics.

Parameters	Mean ± SD/median, *n*%
Dialysis (mon)	50.8 ± 33.7
Age (y)	57.5 ± 14.3
Weight (kg)	55.9 ± 11.2
FGF23 (pg/ml)	3520.4 ± 3678.2
PTH (pmol/l)	59.6 ± 48.3
Calcium (mmol/l)	2.3 ± 0.2
Phosphorus (mmol/l)	2.2 ± 0.4
Serum creatinine (umol/l)	1002.3 ± 254.2
BUN (mmol/l)	26.8 ± 3.8
UA (mmol/l)	453 ± 102.4
Glucose (mmol/l)	7.95 ± 3.41
Hemoglobin (g/l)	109 ± 13.6
ALB (g/l)	40.1 ± 3.3
TG (mmol/l)	1.9 ± 1.2
CHOL (mmol/l)	3.8 ± 1.3
LDL (mmol/l)	2.11 ± 0.68
HDL (mmol/l)	1.07 ± 0.27
BNP (pg/ml)	160.27
Gender (women %)	49 (45.8)
Death (%)	14 (13.0)
Hypertension (yes %)	80 (74.7)
Diabetes (ye s%)	30 (28.0)
Coronary heart disease (yes %)	25 (23.3)
Heart failure (yes %)	52 (48.5)
Stroke (yes %)	8 (7.4)

**Table 2:** The correlation of FGF23 with clinical chemistry parameters (Pearson correlation).

Parameters	FGF23	
	*r*	*p*
Dialysis (mon)	0.07	0.501
Age (y)	−0.44	0.000
Weight (kg)	0.03	0.764
PTH	0.25	0.010
Calcium	0.27	0.005
Phosphorus	0.23	0.017
Serum creatinine	0.19	0.050
BUN	0.18	0.071
UA	0.20	0.042
Glucose	−0.12	0.215
Hemoglobin	0.05	0.587
ALB	0.22	0.023
TG	0.12	0.222
CHOL	0.01	0.899
LDL	0.06	0.546
HDL	0.18	0.065
BNP	−0.13	0.178

**Table 3:** Multivariate linear regression for FGF23.

Independent variables	FGF23		
	*p* value	Coefficients	95.0% confidence interval for *B*
Constant	0.249	−7064.51	−19141.32∼5012.29
Age	0.001	−76.25	−120.17∼ −32.33
PTH	0.010	17.22	4.16∼30.28
Calcium	0.004	4387.78	1470.04∼7305.52
Phosphate	0.990	−8.48	−1338.75∼1321.79
Uric acid	0.136	5.20	−1.66∼12.07
Albumin	0.725	37.47	−172.89∼247.82

**Table 4:** Comparison of the clinical data and biochemical indexes among the different FGF23 level groups.

Items	Group 1, *N* = 26	Group 2, *N* = 25	Group 3, *N* = 27	Group 4, *N* = 29	*p* value
	(3.75–172.03)	(182.13–1146.13)	(1186.17–6314.80)	(6438.10–14610.14)	
Age (y)	61.08 ± 17.28	65.40 ± 13.37	58.37 ± 14.87	46.83 ± 12.48	0.324
Dialysis time (mon)	63.27 ± 38.93	50.16 ± 19.46	66.56 ± 30.22	61.38 ± 29.68	0.137
Hb (g/L)	109.23 ± 15.07	108.32 ± 18.33	110.37 ± 13.69	111.06 ± 13.56	0.847
Alb (g/L)	40.19 ± 3.07	39.66 ± 3.91	40.33 ± 2.68	41.63 ± 2.82	0.596
sCr (umol/L)	944.22 ± 283.99	1021.74 ± 224.36	1059.98 ± 266.39	1072.73 ± 249.21	0.284
UA (mmol/L)	459.25 ± 99.42	437.73 ± 88.65^a^	445.64 ± 125.22	484.86 ± 73.96^a^	**0.038**
Ca (mmol/L)	2.17 ± 0.17	2.18 ± 0.25^a^	2.24 ± 0.22	2.35 ± 0.31^a^	**0.033**
P (mmol/L)	2.00 ± 0.64	2.06 ± 0.50	2.16 ± 0.45	2.27 ± 0.58	0.102
PTH (pmol/L)	46.91 ± 38.09^a^	51.81 ± 41.63	54.78 ± 42.98	77.87 ± 67.36^a^	**0.044**
TG (mmol/L)	1.87 ± 1.26	1.93 ± 1.14	1.75 ± 1.43	2.4 ± 1.38	0.863
CHOL (mmol/L)	3.78 ± 0.84	4.44 ± 2.77	3.89 ± 0.92	4.15 ± 0.75	0.261
HDL (mmol/L)	0.98 ± 0.22^a^	1.13 ± 0.28	1.02 ± 0.21	1.15 ± 0.34^a^	**0.028**
LDL (mmol/L)	2.02 ± 0.76	2.00 ± 0.56	2.12 ± 0.74	2.26 ± 0.19	0.907

*Note.* Boldface represents *P* < 0.05.

**Table 5:** The comparison of clinical cardiac ultrasound parameters among different FGF23 concentration groups.

Parameters (cardiac ultrasound)	Group 1 *N* = 26	Group 2 *N* = 25	Group 3 *N* = 27	Group 4 *N* = 29	*p* value
	(3.75–172.03)	(182.13–1146.13)	(1186.17–6314.80)	(6438.10–14610.14)	
LVE *n* (%)	6 (23.0%)	7 (28.0%)	5 (18.5%)	7 (24.1%)	0.881
RAE *n* (%)	15 (57.6%)	17 (68.0%)	22 (81.4%)	13 (44.8%)	0.035
LEH *n* (%)	15 (57.6%)	13 (52.0%)	19 (70.3%)	13 (44.8%)	0.27
Valvular stenosis *n* (%)	14 (53.8%)	10 (40%)	15 (55.5%)	10 (34.4%)	0.315
LVEF (%)	64.11 ± 10.97	65.28 ± 14.19	64.51 ± 9.01	64.63 ± 10.76	0.985

*Note.* LVE: left ventricular enlargement; RAE: right atrial enlargement; LVH: left ventricular hypertrophy; and LVEF: left ventricular ejection fraction. Boldface represents *P* < 0.05.

## Data Availability

The data used to support the findings of this study are included within the article.

## References

[1] Eckardt K. U., Coresh J., Devuyst O. (2013). Evolving importance of kidney disease: from subspecialty to global health burden. *The Lancet*.

[2] Olauson H., Larsson T. E. (2013). FGF23 and klotho in chronic kidney disease. *Current Opinion in Nephrology and Hypertension*.

[3] Wald R., Sarnak M. J., Tighiouart H. (2008). Disordered mineral metabolism in hemodialysis patients: an analysis of cumulative effects in the hemodialysis (HEMO) study. *American Journal of Kidney Diseases*.

[4] Gutierrez O. M., Mannstadt M., Isakova T. (2008). Fibroblast growth factor 23 and mortality among patients undergoing hemodialysis. *New England Journal of Medicine*.

[5] Yoshiko Y., Wang H., Minamizaki T. (2007). Mineralized tissue cells are a principal source of FGF23. *Bone*.

[6] Erben R. G., Andrukhova O. (2017). FGF23-Klotho signaling axis in the kidney. *Bone*.

[7] Khan A. M., Chirinos J. A., Litt H., Yang W., Rosas S. E. (2012). FGF-23 and the progression of coronary arterial calcification in patients new to dialysis. *Clinical Journal of the American Society of Nephrology*.

[8] Ketteler M., Block G. A., Evenepoel P. (2017). Executive summary of the 2017 KDIGO chronic kidney disease-mineral and bone disorder (CKD-MBD) guideline update: what’s changed and why it matters. *Kidney International*.

[9] Batra J., Buttar R. S., Kaur P., Kreimerman J., Melamed M. L. (2016). FGF-23 and cardio vascular disease: review of literature. *Current Opinion in Endocrinology Diabetes and Obesity*.

[10] Faul C., Amaral A. P., Oskouei B. (2011). FGF23 induces left ventricular hypertrophy. *Journal of Clinical Investigation*.

[11] Scialla J. J., Lau W. L., Reilly M. P. (2013). Fibroblast growth factor 23 is not associated with and does not induce arterial calcification. *Kidney International*.

[12] Streja E., Norris K. C., Budoff M. J., Hashemi L., Akbilgic O., Kalantar-Zadeh K. (2021). The quest for cardiovascular disease risk prediction models in patients with nondialysis chronic kidney disease. *Current Opinion in Nephrology and Hypertension*.

[13] Evenepoel P., Meijers B., Viaene L. (2010). Fibroblast growth factor-23 in early chronic kidney disease: additional support in favor of a phosphate-centric paradigm for the pathogenesis of secondary hyperparathyroidism. *Clinical Journal of the American Society of Nephrology*.

[14] Isakova T., Xie H., Yang W. (2011). Fibroblast growth factor 23 and risks of mortality and end-stage renal disease in patients with chronic kidney disease. *Journal of the American Medical Association*.

[15] Seiler S., Reichart B., Roth D., Seibert E., Fliser D., Heine G. H. (2010). FGF-23 and future cardiovascular events in patients with chronic kidney disease before initiation of dialysis treatment. *Nephrology Dialysis Transplantation*.

[16] Lavi-Moshayoff V., Wasserman G., Meir T., Silver J., Naveh-Many T. (2010). PTH increases FGF23 gene expression and mediates the high-FGF23 levels of experimental kidney failure: a bone parathyroid feedback loop. *American Journal of Physiology—Renal Physiology*.

[17] Koiwa F., Kazama J. J., Tokumoto A. (2005). Sevelamer hydrochloride and calcium bicarbonate reduce serum fibroblast growth factor 23 levels in dialysis patients. *Therapeutic Apheresis and Dialysis*.

[18] Chue C. D., Townend J. N., Moody W. E. (2013). Cardiovascular effects of sevelamer in stage 3 CKD. *Journal of the American Society of Nephrology*.

[19] Soriano S., Ojeda R., Rodriguez M. (2013). The effect of phosphate binders, calcium and lanthanum carbonate on FGF23 levels in chronic kidney disease patients. *Clinical Nephrology*.

[20] Hisatome I., Li P., Miake J. (2021). Uric acid as a risk factor for chronic kidney disease and cardiovascular disease-Japanese guideline on the management of asymptomatic hyperuricemia. *Circulation Journal*.

[21] Schaefer F., Doyon A., Azukaitis K. (2017). Cardiovascular phenotypes in children with CKD: the 4C study. *Clinical Journal of the American Society of Nephrology*.

[22] Leifheit-Nestler M., Grobe Siemer R., Flasbart K. (2016). Induction of cardiac FGF23/FGFR4 expression is associated with left ventricular hypertrophy in patients with chronic kidney disease. *Nephrology Dialysis Transplantation*.

[23] Yamada S., Giachelli C. M. (2017). Vascular calcification in CKD-MBD: roles for phosphate, FGF23, and klotho. *Bone*.

[24] Song T., Fu Y., Wang Y. (2021). FGF-23 correlates with endocrine and metabolism dysregulation, worse cardiac and renal function, inflammation level, stenosis degree, and independently predicts in-stent restenosis risk in coronary heart disease patients underwent drug-eluting-stent PCI. *BMC Cardiovascular Disorders*.

